The article "Using Convolutional Neural Network as a Statistical Algorithm to Explore the Therapeutic Effect of Insulin Liposomes on Corneal Inflammation" was published in 2022. Journal: Comput Intell Neurosci.

# Using Convolutional Neural Network as a Statistical Algorithm to Explore the Therapeutic Effect of Insulin Liposomes on Corneal Inflammation

**DOI:** 10.1155/2022/1169438

**Published:** 2022-07-31

**Authors:** Yukun Liao, Huiting Jiang, Yangrui Du, Xiaojing Xiong, Yu Zhang, Zhiyu Du

**Affiliations:** ^1^Department of Ophthalmology, Second Affiliated Hospital of Chongqing Medical University, Chongqing Medical University, Chongqing, 400010, China; ^2^Chongqing Key Laboratory of Ultrasound Molecular Imaging, Second Affiliated Hospital of Chongqing Medical University, Chongqing Medical University, Chongqing, 400010, China

## Abstract

Aiming at the disadvantages of easy recurrence of keratitis, difficult eradication by surgery, and easy bacterial resistance, insulin-loaded liposomes were prepared, and convolutional neural network was used as a statistical algorithm to build SD rat corneal inflammation model and study insulin-loaded liposomes, alleviating effect on corneal inflammatory structure in SD rats. The INS/PFOB@LIP was developed by means of thin-film dispersive phacoemulsification, its structure was monitored using a transmission electron microscope, particle size and appearance potential were monitored using a Malvern particle sizer, and ultraviolet consumption spectrum was monitored using a UV spectrophotometer. The encapsulation rate, drug loading, and distribution of insulin liposomes in rat corneal inflammatory model were measured and calculated. The cytotoxicity of liposome materials was evaluated by CCK-8 assay, and the toxic effects of insulin and insulin liposomes on cells were detected. The cornea of SD rats was burned with NaOH solution (1 mol/L), and the SD rat corneal inflammation model was created. The insulin liposome was applied to the corneal inflammation model, and the therapeutic effect of insulin liposome on corneal inflammation was evaluated by slit lamp, corneal immunohistochemistry, corneal HE staining, and corneal Sirius red staining. Insulin-loaded liposomes were successfully constructed with an average particle size of (130.69 ± 3.87) nm and a surface potential of (−38.24 ± 2.57) mV. The encapsulation rate of insulin liposomes was (48.89 ± 1.24)%, and the drug loading rate was (24.45 ± 1.24)%. The SD rat corneal inflammation model was successfully established. After insulin liposome treatment, the staining area of corneal fluorescein sodium was significantly reduced, the corneal epithelium was significantly thickened, the content of corneal collagen was increased, the expression of inflammatory factors was significantly reduced, and new blood vessels (corneal neovascularization, CNV) growth was inhibited.

## 1. Introduction

The cornea is a kind of crystal clear tissue, which plays a pivotal role in the improvement of visual function. Considering that the cornea has direct contact with the surrounding space, it also replaces the mechanical protective layer and has an important barrier effect on microorganisms, poisons, and injuries [1]. The cornea is located in the outermost layer of the eye and is highly susceptible to infection. The infection rate of the cornea accounts for 15% of eye injuries, and corneal inflammation is the most common [2]. Various external factors may cause keratitis. It is one of the common eye diseases and one of the major blinding eye diseases in the world. The cornea is located at the front of the eyeball and is in direct contact with the outside world. The clinical manifestations are blurred vision, pain, photophobia and lacrimation, and other stimuli symptoms and obvious vision loss. Ophthalmological examination showed the disappearance of corneal luster, reduced transparency, and ulceration. In severe cases, corneal perforation, intraocular infection, and even blindness may occur. At present, keratitis is divided into infectious, immune, dystrophic, nerve paralysis, and exposure according to the pathogenic cause. Infectious keratitis mostly occurs in the central area of the cornea, while immune keratopathy tends to occur in the peripheral area of the cornea [3].

Insulin (INS) is a small molecule protein with anti-inflammatory, antiapoptotic, and cell growth-promoting effects. It can be used to treat chronic inflammation and promote wound healing. Due to the barrier effect of the tear film and the cornea, the efficiency of drug entry into the eye is extremely low. The liposome (LIP) drug-delivery system can improve drug bioavailability [4]. Liposomes are artificial spherical vesicles composed of single or multiple phospholipid bilayers, with a hydrophilic structure inside and a lipophilic structure outside, similar to cell membranes. Liposomes have complete biodegradability, low toxicity, and high stability, and can also prolong the residence time of encapsulated drugs on the corneal surface through sustained release. They have been used in ophthalmology as drug carriers in the 20th century [5].

Because of its good corneal penetration and biocompatibility, as well as the advantages of targeting and sustained release, it is suitable for applications in the field of ophthalmology. Eye instillation is a commonly used administration method in ophthalmology. Compared with ocular injection, eye drops can reduce the infection risk and economic burden of patients and improve patient compliance. Using liposomes as a carrier can improve the stability, bioavailability, and targeting of insulin on the ocular surface, reduce systemic adverse reactions, and eye irritation, and achieve a sustained release effect [6]. In order to better detect the effect of liposomes on drug loading and cell activity, the method of deep learning is used for relevant statistical analysis. As a common form of deep learning, convolutional neural network is now processing experimental data [7–10] and it is widely used. A convolutional neural network is a multilayer neural network with a deep supervised learning architecture that can be viewed as a combination of two parts: an automatic feature extractor and a trainable classifier. The feature extractor includes convolution filtering and downsampling [11, 12]. The convolution filter kernel on the feature map is usually 3*∗*3, and the downsampling operation after filtering usually has a ratio of 2. The classifier is composed of a fully connected network, and the features learned by the feature extractor will be output by the fully connected layer [13–15]. The purpose of this study was to use convolutional neural network as a statistical algorithm to construct a model of corneal inflammation in SD rats and to explore the therapeutic effect of insulin liposomes on corneal inflammation.

## 2. Materials and Methods

### 2.1. Experimental Drugs

Recombinant human insulin (Beijing Soleibao Technology Co., Ltd.), soybean lecithin (purity ≥99%, Shanghai McLean Biochemical Technology Co., Ltd., China), cholesterol (China Xianruixi Biotechnology Co., Ltd.), perfluorooctane (PFOB, purity ≥99%, USA, Sigma), chloroform (CHCL3, Chongqing Chuandong Chemical Group), methanol (CH3OH, Chongqing Chuandong Chemical Group), and methoxy polyethylene glycol 2000-distearoyl phosphatidylethanolamine were used.

### 2.2. Experimental Apparatus

The experimental instruments used in this experimental study are shown in Table 1.

### 2.3. Experimental Animals

Forty SPF healthy SD rats aged 10 to 12 weeks were selected, and the right eye was taken as the experimental eye, with a body weight of 300 g to 450 g (provided by the Animal Experiment Center of the Chongqing Medical University). Before the experiment, the animals were observed in the animal experiment center for one week, and routine slit lamp examination was performed to exclude diseases related to the ocular surface.

### 2.4. Preparation of Insulin Liposomes

Insulin liposomes were prepared by thin-film dispersion phacoemulsification method. We weighed appropriate amount of soybean lecithin, DSPE-PEG2000, and cholesterol. All three were dissolved in chloroform at a temperature of 50°C and a rotational speed of 130 rpm. The organic solvent was evaporated to dryness under the swirl, so that a uniform film was formed in the round-bottomed flask, and then the buffer reagent was added, and the treatment was performed by shaking and washing the film, and ultrasonically emulsified for 30 W 1 min to form a W/O emulsion. The emulsion was added to the film eluent, and sonicated for 45 W 3 min to obtain nanoparticle liposomes. Then, centrifuge at 6000 rpm/min for 5 min, remove the supernatant, collect the precipitate, store at 4°C, low temperature, and protect from light for later using.

### 2.5. Characterization Assay of Insulin Liposomes

Particle size and potential: take 100 *µ*L of insulin diluted hydrochloric acid solution, dissolve it in triple distilled water, and measure the particle size and Zeta potential of INS/PFOB@LIP with a Malvern particle size. Encapsulation efficiency and drug loading: prepare a certain amount of insulin liposomes, and measure the encapsulation efficiency and drug loading of the drug by the demulsification method. The calculation formula is as follows:

(1) $$\begin{array}{c} \phi =\frac{P_{\text{in}}}{P_{\text{all}}}\times 100\%, \end{array}$$

(2) $$\begin{array}{c} \eta =\frac{P_{\text{in}}}{Z_{\text{all}}}\times 100\%, \end{array}$$

where *Φ* represents the insulin encapsulation rate; *P*_in_ represents the drug loading; *P*_all_ represents the total input amount; *η* represents the insulin drug loading rate; and *Z*_all_ represents the total amount of liposomes.

### 2.6. Liposome Distribution and Animal Model Establishment

In a dark environment, the corneal inflammation model rats were instilled with DiI-labeled insulin liposomes. After 2 h, the corneas were removed, and 10 *µ*m frozen sections were made. Insulin immunofluorescence staining was observed and photographed under a fluorescence microscope.

40 SD rats (provided by the Animal Experiment Center, Chongqing Medical University, on behalf of them), weighing 300 g to 450 g, were randomly divided into normal saline group (NS group), liposome empty sphere group (PFOB@LIP), insulin group (INS), and insulin liposome group (INS/PFOB@LIP), 10 in each group. Three days before modeling, rats were given 30 *µ*L/time of levofloxacin eye drops in cornea and conjunctival sac of both eyes, three times a day for 3 days. The rats were anesthetized by intraperitoneal injection of 4 mL/kg ketamine solution (100 mg/mL), and 30 *µ*l of lidocaine hydrochloride eye drops was administered. A circular filter paper with a diameter of 3 mm infiltrated with NaOH solution was placed in the center of the cornea of the right eye of the rat for 40 s, the cornea and conjunctival sac were washed with a large amount of normal saline for 3 minutes, and the left eye was left without any treatment to establish a control experiment of corneal epithelial cell inflammation model. We used NS, PFOB@LIP, INS, and INS/PFOB@LIP (the concentration of liposomes in PFOB@LIP and INS/PFOB@LIP is 400 *µ*g/mL, and the concentration of INS is 200 *µ*g/mL) in the right eye, respectively, 30 *µ*L, once in the morning, noon, and night, for 14 days.

### 2.7. Evaluation of the Therapeutic Effect of Keratitis

At 1, 3, 7, and 14 days after the corneal epithelial cells appeared obvious inflammation, the cornea and new blood vessels were observed and photographed under white light and no red light using a slit lamp. 2 *µ*L of 1% fluorescein sodium dye solution was given to stain the cornea, and the excess dye solution is rinsed with normal saline. The cornea was observed and photographed under cobalt blue light using a slit lamp. Referring to the literature [6], the cornea is divided into 4 parts by the horizontal and vertical axes, and Image-*J* software is used to analyze and calculate the area of corneal neovascularization of each part and sum up 3 rats were randomly selected from each group at each time point, sacrificed by cervical dislocation, and corneal tissue was harvested for tissue fixation, embedding, and sectioning. To detect the uptake of liposomes by cells, the red cell membrane fluorescent probe DiI was loaded into the liposomes as a fluorescent dye. After 24 h of incubation, paraformaldehyde was fixed and HE staining was used to observe epithelial cells and fibrous tissue and the number of inflammatory cells. The arrangement and content of collagen fibers were observed by sirius scarlet staining. Immunohistochemical staining was used to detect the protein expressions of CD31, IL-1*β*, and TNF-*α*. Image-J software was used to analyze the positive reaction sites in the photographs, and the relative optical density was measured.

### 2.8. Statistical Analysis Based on Convolutional Neural Network Algorithm

In order to better detect the effects of insulin liposomes on drug loading, cell activity, and the therapeutic effect of keratitis, a deep learning method was used to conduct relevant statistical analysis [16, 17]. The convolutional neural network algorithm is one of the most important frameworks in deep learning. It can make good use of the prior information of “space-time locality” in the data, so as to achieve the purpose of enabling the network to remember past time information, so that the network can not only realize the connection from bottom to top (input-output), but also realize the information transmission and recording from left to right (time *t* to time *t* +  1).

Convolutional neural network is constructed by imitating the visual perception mechanism of biology, which can perform supervised learning and unsupervised learning. Small computational effort for grid-like topology features, such as modeling insulin absorption and depletion, with stable effects and no additional feature engineering requirements on the data [18–21]. Therefore, the use of the convolutional neural network algorithm can more accurately analyze the data collected from the experiment. The statistical data are expressed as the mean ± standard deviation, which is statistically significant. The specific algorithm flow is as follows.

#### 2.8.1. Forward Propagation

*(1) Convolutional Layer*. The network search data are two-dimensional feature data. After the input data and the filter are convolved, the local features of the data are extracted. In this paper, *X*_*j*_^*l*^ is used to represent the output of the 1th channel of the convolutional layer, *W*_*ij*_^*l*^ is the weight vector of the *1*th channel of the convolutional layer, *b*_*j*_^*l*^ is the bias vector of the layer, and *M*_*j*_ is the receptive field of the convolution kernel on the input data, “*∗*” represents the convolution operation, *f*(*∗*) is the activation function, the process of extracting features is shown in [22, 23]

(3) $$\begin{array}{c} z_{j}^{l}=\sum_{i\in M_{j}}X_{i}^{l-1}*W_{ij}^{l}+b_{j}^{l},\\ X_{j}^{l}=f\left(z_{j}^{l}\right). \end{array}$$

In the convolution layer, a convolution kernel is only locally connected to the input data and has nothing to do with other data, reducing irrelevant connections, which is the local receptive field; at the same time, this convolution kernel uses the same volume on one channel of the data. The product kernel performs feature mapping and reduces the number of parameters, which is called weight sharing. These two characteristics are one of the cores of the simplified operation of convolutional neural network.

*(2) Downsampling Layer*. Downsampling the data can reduce the amount of data processing while retaining the useful information of the data, which is another major feature of the convolutional neural network to reduce parameter calculation [24–26]. The downsampling generally uses a 2*∗*2 window. If it is a maximum pooling layer, the maximum value of the 2*∗*2 numbers is taken; if it is an average pooling layer, the average of these 4 numbers is taken. *X*_*j*_^*l*^ represents the feature of the *j*-th channel in layer *l*, *β*_*j*_^*l*^ is the weight, and *b*_*j*_^*l*^ is the bias. *down* ( ) represents downsampling, *f* ( ) is the activation function, then the principle of the downsampling layer is as follows:

(4) $$\begin{array}{c} z_{j}^{l}=\beta_{j}^{l}\text{ down }\left(X_{j}^{l-1}\right)+b_{j}^{l},\\ X_{j}^{l}=f\left(z_{j}^{l}\right). \end{array}$$

*(3) Fully Connected Layer*. The data passing through the convolutional layer is flattened into a one-dimensional vector, and then enters the fully connected layer for classification or regression. The calculation of the fully connected layer is shown in (2). In the sales forecast, it is a regression problem, and the output is a real number, so the loss function adopts MSE (mean square error). The calculation formula of MSE is shown in (4), where ${\hat{y}}_{i}$ represents the predicted value, *y*_*i*_ represents the real value, and *m* is the number of samples [27, 28].

(5) $$\begin{array}{c} X^{l}=f\left(W^{l}X^{l-1}+b^{l}\right),\\ \text{MSE}=\frac{1}{m}\sum_{i=1}^{m}{\left({\hat{y}}_{i}-y_{i}\right)}^{2}. \end{array}$$

#### 2.8.2. Backpropagation

In the forward propagation phase, the loss of the model is obtained in each round of iteration. In the back propagation phase, the loss is backpropagated through the gradient descent method to update the weights and biases of each layer of the convolutional neural network. Through parameter update, the loss of the model no longer decreases, then the requirement is met. The main reference for backpropagation of convolutional neural networks is [29, 30].

*(1) Convolutional Layer*. Since the next layer of the convolutional layer is usually a downsampling layer, the sensitivity of the downsampling layer needs to be used to represent the sensitivity of the convolutional layer during backpropagation. For example, if the maximum pooling layer is used, the size of the pooling area is 2*∗*2, each value of the *l* +  1 layer corresponds to the 2*∗*2 area of the lth layer, and the up-operation puts each value of the *l*  +  1 layer into the Return to the position of the original maximum value of this 2*∗*2 area and adds 0 to other positions. *δ* represents the Hadamard product, representing the multiplication of the corresponding elements of the matrix, and then the sensitivity of the convolutional layer is [31, 32]

(6) $$\begin{array}{c} \delta_{j}^{l}=\beta_{j}^{l+1}\left(f^{\prime }\left(z_{j}^{l}\right)\circ \text{ up }\left(\delta_{j}^{l+1}\right)\right). \end{array}$$

When deriving the parameters of the convolution kernel, it is necessary to consider the input features multiplied by the convolution kernel. *x*_*u*+*i*−1, *y*+*j*−1_^*l*−1^ is the part that is multiplied by *W*_*ij*_^*l*^ input elements, *η* is the learning rate, and then the weights of the convolutional layers are updated as follows:

(7) $$\begin{array}{c} W_{ij}^{l}=W_{ij}^{l}-\eta \sum_{u}\sum_{v}\left(\delta_{uv}^{l}x_{u+i-1,\;v+j-1}^{l-1}\right). \end{array}$$

Since each output value of the channel is related to the bias term, the gradient of the bias term is the sum of the sensitivity elements of the channel and the bias term is updated as follows [33]:

(8) $$\begin{array}{c} b_{j}^{l}=b_{j}^{l}-\eta \sum_{u,v}{\left(\delta_{j}^{l}\right)}_{u,v}. \end{array}$$

*(2) Downsampling Layer*. When the lth layer is a downsampling layer, assuming that the *l* + 1th layer is a convolutional layer, the sensitivity of the next layer is used to represent the sensitivity of the previous layer, and the calculation is as follows [34]:

(9) $$\begin{array}{c} \delta_{j}^{l}=\delta^{l+1}*\text{ rot }180\left(W_{j}^{l}\right)\circ f^{\prime }\left(z_{j}^{l}\right). \end{array}$$

*rot*180 (*W*_*j*_^*l*^) means that the convolution kernel is rotated by 180°, and *δ*^*l*^ ^+^ ^1^ needs to be filled with 0 s on its boundary, so that the size is the same as *z*_*j*_^*l*^. The update of the bias term and weight is shown in the following equations [35]:

(10) $$\begin{array}{c} b_{j}^{l}=b_{j}^{l}-\eta \sum_{u,v}{\left(\delta_{j}^{l}\right)}_{u,v}, \end{array}$$

(11) $$\begin{array}{c} \beta_{j}^{l}=\beta_{j}^{l}-\eta \sum_{u,v}{\left(\delta_{j}^{l}\circ \text{ down }\left(X_{j}^{l-1}\right)\right)}_{u,v}. \end{array}$$

## 3. Results

### 3.1. Effects of Insulin and Insulin Liposomes on Corneal Cell Viability

The cytotoxicity of liposome materials was evaluated by CCK-8 assay, and the toxic effects of insulin and insulin liposomes on cells were detected. The cytotoxic effects of liposomal materials were investigated using corneal cells.  Figure 1 shows the viability of cells after insulin, blank liposome, and insulin liposome treatment. The cells treated with blank liposomes still had a cell viability of more than 90% after being placed for 400 h, indicating that the liposome material has high biocompatibility and no obvious cytotoxicity.

The results show that INS/PFOB@LIP can significantly increase the cell activity of corneal cells for 20 h, so this study selects insulin liposomes for follow-up experiments.

### 3.2. Physicochemical Properties, Encapsulation Efficiency, and Drug Loading Capacity of Liposomes

We dissolve PFOB@LIP and INS/PFOB@LIP in PBS to prepare 400 *µ*g/mL 2 mL. The INS solution (200 *µ*g/mL 2 mL) is colorless and transparent, the PFOB@LIP and INS/PFOB@LIP suspensions are milky white, and the INS/PFOB@LIP suspension is dark. Transmission electron microscopy showed that INS/PFOB@LIP had a relatively uniform and consistent spherical appearance, the liposome was a shell-core structure, and a phospholipid bilayer could be observed (Figure 1(a)). The average particle size of PFOB@LIP is (105.39 ± 2.83) nm, and the average particle size of INS/PFOB@LIP is (130.69 ± 3.87) nm (Figures 2(b) and 2(c). The Zeta potentials of PFOB@LIP and INS/PFOB@LIP were (−10.03 ± 1.27) mV and (−38.24 ± 2.57) mV, respectively (Figure 1(d)) (*P* < 0.001, the difference was statistically significant). According to the physical and chemical properties of INS, it can be expressed by the following linear regression equation: *Y* = 0.01476 × *X*−0.1203, *R*^2^ = 0.9854; the encapsulation efficiency and drug loading of insulin INS are calculated as (48.89 ± 1.24)% and (24.45 ± 1.24)%.

### 3.3. Distribution of Liposomes in Rats

After 4 h, the frozen sections of the cornea were taken out in batches for testing. The results showed that the cornea had a strong fluorescent signal, indicating that the insulin liposomes had entered the eye and were diffusely distributed. To more accurately measure the distribution of liposomes in rats, the uptake of fluorescent liposomes by corneal epithelial cells was observed by confocal laser microscopy. It can be seen that the fluorescent liposomes in the nuclei and corneal epithelial cells gradually increased, as shown in Figure 3. This indicated that the uptake of insulin liposomes by corneal epithelial cells increased with time, indicating that corneal epithelial cells had strong uptake ability to liposomes.

### 3.4. Evaluation of the Therapeutic Status of Rat Corneal Inflammation

In order to more accurately analyze the therapeutic effect of insulin liposome on corneal inflammation, statistical analysis was done using convolutional neural network. First, the percentage of corneal epithelial defect area is extracted separately, the percentage of corneal epithelial defect area, NS, PFOB@LIP, INS, and INS/PFOB@LIP is brought into the convolutional neural network statistical analysis model, and the results are shown in Figure 4(a). As can be seen from Figure 4(a), in 1 d–7 d, the corneal epithelial defect area gradually decreased, and the percentage of corneal epithelial defect area at 7 days was (34.49 ± 0.98)% in the NS group; (32.43 ± 0.18)% in the PFOB@LIP group; and (0.54 ± 0.4)%; INS/PFOB@LIP group was (0 ± 0)%, and INS group and INS/PFOB@LIP group basically healed. INS/PFOB@LIP compared with each group, the difference was statistically significant (*P* < 0.01). On the 7-th day, the new blood vessels in each group exceeded the cornea and tended to invade the center of the cornea. The new blood vessels were small, pale, sparse, and brush-shaped. On the 14-th day, the new blood vessels in each group grew towards the burn area, the blood vessels gradually thickened and denser, and the growth of INS/PFOB@LIP blood vessels was the slowest. From 7 d to 14 d, the new blood vessels increased in each group, and the area of new blood vessels in the INS and INS/PFOB@LIP groups was significantly smaller than that in the other groups.

Secondly, the recalculated area percentage of new blood vessels in each group after 7 days and 14 days, NS, PFOB@LIP, INS, and INS/PFOB@LIP were brought into the convolutional neural network statistical analysis model, and the results are shown in Figure 4(b). As shown in Figure 4(b), the area of new blood vessels in the INS/PFOB@LIP group was smaller than that in the other groups, and the difference was statistically significant (*P* < 0.05). Through daily inspection, it was found that the corneal epithelium of each group had different degrees of defects on the 1st and 3rd day after the cornea of the rats appeared inflammation, which did not reach the normal cell coverage of 6–8 layers, the arrangement of collagen fibers was loose and disordered, and a large number of inflammatory cells were infiltrated. At 7 d, the corneal epithelium of NS and PFOB@LIP was still defective and the tissue structure was disordered. The epithelial cells of INS and INS/PFOB@LIP basically reached 5–6 layers. In the four groups, the inflammatory cells and corneal thickness reached the peak value, and the formation of neovascular cavity was seen in the stromal layer. On the 14th day, the inflammatory cells in the four groups were reduced, the corneal epithelial cells reached 6–7 layers, and a large number of new blood vessels were formed, red blood cells infiltrated in the lumen, and the corneal tissue structure tended to be neat. After 14 days, the rat corneal cells were detected, and it was found that in the INS/PFOB@LIP group, the collagen fibers in the cornea were densely arranged and not neatly arranged, while the collagen fibers in the other three groups were thick, abundant, criss-cross, loose, and disordered. Histochemical staining was used to observe the growth of corneal neovascularization and inflammatory infiltration by vascular endothelial cell marker CD31, inflammatory cell markers IL-1*β,* and TNF-*α*. On the 14-th day, NS, PFOB@LIP, and INS showed a large amount of angiogenesis and a large number of inflammatory cells infiltration. The relative optical density of each cytokine was detected by immunohistochemical method on 14 days, the average optical density of the blank control group was used as the reference, and the parameter was 1. The relative optical density of each group is shown in Figure 4, and the difference between each group was statistically significant (*p* < 0.05):

- *P* < 0.01, compared with INS/PFOB@LIP group. In each group, the area of corneal epithelial inflammation gradually decreased for 7 days, INS and INS/PFOB@LIP healed completely, and INS/PFOB@LIP recovered the fastest.
- *P* < 0.05, compared with the INS/PFOB@LIP group. The area of neovascularization in each group increased at 14 days, and the area of neovascularization in the INS/PFOB@LIP group was the least.

## 4. Conclusion

We successfully prepared liposomes loaded with PFOB and INS by thin-film dispersion phacoemulsification. The prepared liposomes had a typical shell-core structure, and insulin and perfluorooctane were encapsulated in the phospholipid membrane layer. Through DiI staining of liposomes, it can be seen that liposomes can enter and diffusely distribute in the eye, so as to achieve better therapeutic effect, establish an SD rat model of corneal inflammation, and observe the therapeutic effect of INS/PFOB@LIP on alkali burns. In order to more accurately analyze the therapeutic effect of insulin liposomes on corneal inflammation, the convolutional neural network statistical analysis method was used. The percentage of corneal epithelial defect area, percentage of new blood vessel area, NS, PFOB@LIP, INS, and INS/PFOB@LIP in each group were included in the convolutional neural network statistical analysis model, and the convolutional neural network statistical analysis algorithm showed the treatment effect. After 7 d of treatment, compared with NS, PFOB@LIP, and INS, the corneal epithelium of INS/PFOB@LIP was almost completely healed with minimal neovascularization. After 14 days of treatment, compared with NS, PFOB@LIP, and INS, the growth rate of new blood vessels in INS/PFOB@LIP group was the slowest. It can be seen that INS/PFOB@LIP has good anti-inflammatory and antiangiogenesis effects.

At different time intervals, the occurrence and development of corneal epithelial defect, corneal edema, corneal opacity, and corneal neovascularization of NS, PFOB@LIP, INS, and INS/PFOB@LIP were observed under slit lamp. After 7 days of treatment, compared with NS, PFOB@LIP and INS, the corneal epithelium of INS/PFOB@LIP was almost completely healed with minimal neovascularization. After 14 days of treatment, compared with NS, PFOB@LIP, and INS, the growth rate of new blood vessels in the INS/PFOB@LIP group was the slowest. The results of HE staining, Sirius red, and immunohistochemistry showed that after topical application of INS/PFOB@LIP eye drops, the inflammatory factors in the INS/PFOB@LIP group were lower than those in the NS, PFOB@LIP, and INS groups, and the collagen fibers were densely arranged and there were followed by the other three groups. Using CD31 to label neovascular endothelial cells, it could be observed that the number of neovascularization in INS/PFOB@LIP was significantly lower than that in NS, PFOB@LIP, and INS groups.

In conclusion, insulin liposome INS/PFOB@LIP can significantly improve the cell activity of corneal cells for 20 h. The convolutional neural network algorithm was used to carry out the relevant statistical analysis, and the experimental data was analyzed by the algorithm. It can be seen that after the insulin liposome INS/PFOB@LIP treatment, the symptoms of keratitis were alleviated, the INS/PFOB@LIP corneal epithelium was basically completely healed, and the new angiogenesis was the least, and compared with other experimental control groups, the INS/PFOB@LIP group had lower inflammatory factors than NS, PFOB@LIP, and INS groups, and the differences were statistically significant (*P* < 0.01), demonstrating that insulin liposomes can be used as potential therapeutics for corneal inflammation.

## Figures and Tables

**Figure 1:** The effects of INS, PFOB@LIP, and INS/PFOB@LIP on corneal cell viability.

**Figure 2:** (a) TEM of INS/PFOB@LIP (50 *µ*g/mL). (b) Particle size distribution of PFOB@LIP. (c) Particle size distribution of INS/PFOB@LIP. (d) Zeta potential maps of PFOB@LIP and INS/PFOB@LIP.

**Figure 3:** (a) Blue represents DAPI. (b) Green represents insulin. (c) Red represents liposomes. (d) Fluorescence image of cornea after 2 hours (×400).

**Figure 4:** (a) 7 days comparison of corneal inflammation area; (b) 14 days comparison of new blood vessel area.

**Table 1:** Instruments required for the experiment.

Experimental instrument name	Company
Rotary evaporator	Shanghai Yarong Biochemical Instrument Factory
Sonicator	United States, Sonics
37°C cell incubator and light microscope	Olympus Corporation
Dragonfly 200 high-speed confocal imaging platform	Oxford Instruments Technology Ltd
4°C centrifuge	Thermofisher Corporation
Transmission electron microscope	TEM, Japan, HiTachi

## Data Availability

The dataset can be accessed upon request to the corresponding author.
